# Excimer Laser Corneal Refractive Surgery in the Clinic: A Systematic Review and Meta-analysis

**DOI:** 10.1155/2022/7130422

**Published:** 2022-06-15

**Authors:** Huang Zhang, Mingming Li, Zhimin Cen

**Affiliations:** Department of Ophtalmology, Zhongshan Torch Development Zone People's Hospital, Zhongshan 528437, Guangdong Province, China

## Abstract

**Objective:**

To systematically evaluate the efficacy, safety, recovery speed, and long-term visual quality of excimer laser corneal refractive surgery and to provide evidence-based medicine for the promotion and use of excimer laser corneal refractive surgery.

**Methods:**

Randomized controls on excimer laser refractive surgery in Web of science, PubMed, EMBASE, ScienceDirect, Cochrane Library, China Knowledge Network (CNKI), China VIP Database, Wan Fang Database, and China Biomedical Literature Database (CBM) were searched by the computer. Randomized controlled trial (RCT) data were extracted independently by two researchers, and the risk of bias of each included RCT was assessed according to the Cochrane Handbook 5.1.0 criteria. Meta-analysis of the collected data was performed using RevMan5.4 statistical software.

**Results:**

In the end, 9 high-quality literatures were included, with a total of 4366 samples, and meta-analysis was used. There was no significant difference in uncorrected visual acuity WMD after excimer laser keratorefractive surgery, but there was a statistically significant difference in WMD in the safety of excimer laser keratorefractive surgery. The results of uncorrected visual acuity (close) indicated the following: Chi^2^ = 13.56, DF = 5, *P* = 0.02, and I^2^ = 100%; the results of uncorrected visual acuity (distance) indicated the following: Chi^2^ = 34.44, DF =5 (*P* < 00000), and I^2^ = 85%; the results of best corrected visual acuity (myopia) indicated the following: Chi^2^ = 0.65, DF = 3, *P* = 088 > 0.05, and I^2^ = 0%; the results of best corrected visual acuity (hyperopia) indicated the following: Chi^2^ = 1.80, DF = 3, *P* = 0.61 > 0.05, and I^2^ = 0%.

**Conclusion:**

Excimer laser corneal refractive surgery is safe and effective, with faster recovery and better long-term visual acuity treatment effect. However, more studies and follow-up with higher methodological quality and longer intervention time are needed for further validation.

## 1. Introduction

According to statistics, 300 million people in China suffer from myopia, accounting for about 30% of the total myopia in the world [1]. According to the survey, the worldwide incidence of myopia in children is increasing year by year, seriously endangering the health of children [2]. In the mid-1970s, the rate of myopia among children in most countries was low, accounting for about 15% to 20%. But now, there is a gradual upward trend from small towns, medium-sized cities to big cities, and it is obviously developing from the old age group to the younger age group. In 2000, the results of the fourth national physical health survey of students were jointly organized by the Ministry of Education, the Ministry of Health, and the Ministry of Science and Technology [3]. The myopia rate of students all over the world remains high, including 20.23% for primary school students and 48.18% for junior high school students. The myopia rate of senior high school students is 71.29%, and that of college students is 73.01%. Another survey of senior high school students in four cities shows that among more than 10,000 primary and secondary school students, myopia accounts for 70% to 80% [4]. The incidence of myopia rose from about 15% in the 1970s to 55% in the late 1990s, and even reached about 80% [5]. In the 1990s, the incidence of myopia among high school students in big cities in some developed countries was close to 50% to 60% [6]. Thus, it can be seen that the incidence of myopia is rising rapidly all over the world. Now is the time for the whole society to pay attention and take measures. Myopia is the most common eye disease in the world. With the development of modern social sciences and the changes of people's living and learning conditions and lifestyle, the incidence of myopia is increasing day by day, and the incidence of myopia in children and adolescents is also in advance. Farewell to myopia has become a dream in the hearts of myopic patients [7].

Excimer laser corneal refractive surgery uses excited Argon Fluoride (ArF) gas to release high-energy photons, that is, ultraviolet light with the wavelength of 193 nm [8]. This laser can separate the structural bonds in the corneal tissue, accurately produce light cutting effect, remove the corneal tissue by vaporization, and then change the curvature of the corneal surface to achieve the purpose of refractive correction. Trokel adopted excimer laser in keratectomy in 1983. Since Seiler first used excimer laser keratectomy (PRK) to correct myopia in 1989, excimer laser corneal refractive surgery has been rapidly popularized and developed all over the world [9]. PRK was first introduced and carried out in Beijing Tongren Hospital and Union Hospital in 1993 and has been rapidly popularized in major cities throughout the country in recent years [10]. Especially in the past decade, excimer laser corneal refractive surgery has experienced a process of development, improvement, and maturity from equipment to technology. Excimer laser technology has developed from large light spot cutting and multi-area cutting to the current “flying spot scanning” cutting technology. Lamellar keratectomy machine has developed from manual technology to fully automatic technology. In recent years, with the application of wavefront technology and aspheric cutting technology, excimer laser corneal refractive surgery has entered a new stage of development [11]. It has experienced from the corneal surface to the deep part and then returned to the corneal surface, forming the development pattern of the coexistence of deep corneal refractive surgery represented by LASIK and surface corneal refractive surgery represented by the Epi-LASIK in the next few years [12]. Excimer laser corneal refractive surgery has been developed rapidly for more than ten years, and its short-term effect has been fully affirmed. However, its long-term effect, especially the long-term effect of more than 10 years, is the concern of the majority of ophthalmologists and patients [13]. In this study, the author conducted a meta-analysis on the efficacy, safety, recovery speed, long-term visual quality evaluation, and clinical value of excimer laser corneal refractive surgery, in order to provide relevant reference for patients undergoing excimer laser corneal refractive surgery.

## 2. Research Contents and Methods

### 2.1. The Sources and Retrieval Methods of Documents

Web of science, PubMed, EMBASE, ScienceDirect, Cochrane Library, China knowledge Network (CNKI), China VIP database, Wan Fang database, and China Biomedical Literature Database (CBM) were searched by the computer, and the relevant journals, conference papers, and degree papers were searched. With the method of literature review, the data about the effect, safety, recovery speed, and long-term visual quality of excimer laser corneal refractive surgery in China were collected. Literature retrieval was conducted in the way of free words and subject words, with the keywords of excimer laser corneal refractive surgery, surgical effect, safety, recovery speed, and long-term visual quality from January 2010 to December 2021.

### 2.2. Literature Inclusion Criteria and Exclusion Criteria

#### 2.2.1. Literature Inclusion Criteria

The inclusion criteria are as follows: (1) randomized controlled or observational study; (2) age ≥18 years old; (3) high refractive error, preoperative equivalent spherical refraction ≤-6.00D; (4) no corneal abnormality, elevated intraocular pressure, retinal hole, history of uveitis, diabetes, and autoimmune diseases; (5) excimer laser corneal refractive surgery; and (6) the outcome index should include uncorrected visual acuity (UCVA), BCVA, complications, the number of secondary operations, and the difference between postoperative equivalent spherical lens and expected diopter.

#### 2.2.2. Literature Exclusion Standard

The exclusion criteria are as follows: (1) Literature types are reviews, case reports, self-control design studies, abstracts, and conferences; (2) age <18 years old; (3) incomplete literature data; (4) non-Chinese literature; and (5) patients with moderate myopia (preoperative equivalent spherical diopter is -3.00D to -6.00D).

### 2.3. Quality Evaluation and Data Extraction

Literature screening was completed by two researchers independently. The missing data were linked to the author of the original study, and differences were discussed with a third researcher. Collect all the relevant literature according to the retrieval method, and gradually determine the research included in the quantitative analysis.

Data extraction are as follows: (1) the name, research type, sample size, and follow-up time of the first author and (2) the average preoperative equivalent spherical lens, the range of equivalent spherical lens, the type of operation, and the type of ametropia.

### 2.4. Statistical Processing

ReviewManager5.3 software was adopted to process the data. The combined effect of continuous data was presented by mean difference and 95% confidence interval (CI), and the combined effect of classified data was expressed by relative risk (RR) and 95% CI. The heterogeneity among the literatures was tested by I^2^ test. If I^2^ < 50%, the fixed effect model is adopted for analysis; otherwise, the random effect model is adopted. In order to test the reliability of the results, sensitivity analysis was carried out. The difference exhibited statistically significant (*P* < 0.05).

## 3. Results and Analysis

### 3.1. The Results of Literature Retrieval and the Basic Situation of Literature Inclusion

418 articles were retrieved through computer database; 165 articles were obtained after eliminating repeated studies; 87 articles were obtained from preliminary reading of titles and abstracts; and 25 articles were included after excluding irrelevant studies, reviews, case reports, and no control literature. Then, read the full text in detail, excluding 16 articles with incomplete data and no main outcome indicators, and finally include 9 high-quality literatures [14–22]. A total of 4366 samples were analyzed by meta. The basic features included in the literature are indicated in Table 1.

### 3.2. Evaluation of the Quality of the Methodology Included in the Literature

The nine literatures included in this meta-analysis reported the baseline situation of patients, and the nine studies included gave detailed intervention measures. None of the 9 articles gave a detailed description of the blind method and the number and reasons of those who lost follow-up or withdrew. The evaluation of literature quality can be noticed in Figures 1 and 2.

### 3.3. Meta-analysis Results

#### 3.3.1. Surgical Effect and Recovery Speed

The results of excimer laser corneal refractive surgery in 4366 samples from 9 literatures were analyzed by meta. The results of heterogeneity test indicated that the postoperative naked visual acuity was Chi^2^ = 6.17, DF = 3, *P* = 0.10 > 0.05, and I^2^ = 51%. This indicated that there was obvious heterogeneity among the included research data, and the combined effect size WMD was analyzed by random effects model. According to the analysis in Figure 3, the combined effect size WMD test is *Z* = 0.30 (*P* = 0.77). Preoperative uncorrected visual acuity is as follows: Chi^2^ = 24.33, DF = 2, *P* < 0.0001, and I^2^ = 92%, indicating that there is obvious heterogeneity among the included research data and the combined effect dose WMD was analyzed by fixed effect model. Through the analysis of Figures 4 and 3, it can be concluded that there is no statistical difference in the WMD of naked visual acuity after excimer laser corneal refractive surgery, indicating that the effect and recovery speed of excimer laser corneal refractive surgery are satisfactory.

#### 3.3.2. Security

Through a meta-analysis of the safety of excimer laser keratorefractive surgery in 4366 samples of 9 included literature studies, the results of heterogeneity test indicated the following: Chi^2^ = 20.03, DF = 2, *P* = <0.0001, and I^2^ = 90%, indicating that there is obvious heterogeneity among the included research data. From the analysis of Figure 5, it can be noticed that the WMD of the safety of excimer laser corneal refractive surgery is statistically different, and the 95% confidence level of the WMD falls below the horizontal line. On the right side of the invalid line, it shows that the use of excimer laser corneal refractive surgery is safe.

#### 3.3.3. Long-Term Visual Quality

Through the study of 9 articles, a total of 4366 samples were studied. The long-term visual quality of excimer laser corneal refractive surgery was analyzed by meta. Naked visual acuity (close) is as follows: Chi^2^ = 13.56, DF = 5, *P* = 0.02, and I^2^ = 100%. It shows that there is obvious heterogeneity among the included research data. The combined effect size WMD was analyzed by random effects model, and the test of combined effect size WMD was *Z* = 12.18 (*P* < 0.00001) (see Figure 6). The results of uncorrected visual acuity (distance) indicated the following: Chi^2^ = 34.44, DF = 5 (*P* < 00000), I^2^ = 85% (Figure 7); the results of best corrected visual acuity (myopia) indicated the following: Chi^2^ = 0.65, DF = 3, *P* = 088 > 0.05, and I^2^ = 0%. It shows that there is obvious heterogeneity among the included research data. The combined effect size WMD was analyzed by random effects model, and the combined effect size WMD test was *Z* = 10.96 (*P* < 0.00001), as indicated in Figure 8; the best corrected visual acuity (far) is as follows: Chi^2^ = 1.80, DF = 3, pendant 0.61 > 0.05, and I^2^ = 0%. It shows that there is obvious heterogeneity among the included research data, the combined effect size WMD was analyzed by random effects model, and the test of combined effect size WMD was *Z* = 10.01 (*P* < 0.00001), as indicated in Figure 9. It is considered that the long-term (three years after surgery) visual quality of excimer laser keratorefractive surgery is better.

## 4. Analysis and Discussion

With the progress of scientific and technological information, the group and frequency of computer users are increasing day by day, and the number of myopic patients is also increasing [22]. At present, the main ways to treat myopia are frame glasses, corneal contact lens, and refractive surgery. The progress of society has led to the improvement of people's demand for quality of life, and the desire of myopic patients to remove their glasses is becoming more obvious. More people are willing to choose refractive surgery to treat myopia. In the refractive system of the eye, the corneal refractive power is the largest, with an average of 43.0D, accounting for 74% of the total diopter of the eyeball, so as long as the corneal diopter is slightly reduced, the refractive power of the whole eyeball can be effectively corrected. And the cornea is located on the surface of the eyeball, so the operation is safe and easy to operate [23]. Corneal refractive surgery is the main surgical method for the treatment of myopia. Excimer laser, which originated in early 1970, is an excited dimer laser, which is a combination of compressed inert gas and halogen gas and excited by external energy to form an extremely unstable compound dimer excimer laser [24]. In the past ten years, laser in situ keratomileusis (LASIK), laser epithelial keratomileusis (LASEK), epipolis laser in situ keratomileusis (Epi-LASIK) and intra-laser assisted laser in situ keratomileusis (Intra-LASIK) have appeared successively in excimer laser in situ keratomileusis and then returned to the corneal surface to form the development pattern of the coexistence of deep corneal refractive surgery represented by LASIK and surface corneal refractive surgery represented by Epi-LASIK in the next few years [25, 26].

In the early stage of the development of excimer laser corneal refractive surgery technology, the excimer laser therapeutic instruments produced by most manufacturers adopted the wide-band cutting method of large light spot [26]. This large light spot technology often leads to the following problems: central island effect, corneal opacity, and large light spot treatment, which determines in principle that there are certain limitations when treating hyperopia and astigmatism. In order to overcome the shortcomings of large spot technology, excimer laser therapeutic instruments mostly use small spot (<2 mm) flying spot scanning technology, pulse frequency 50~200 Hz is different, scanning time is shorter, and the cutting area is smoother. The position of each laser spot on the cornea is random, and the superposition of all the light spots can obtain an ideal distribution of light spots on the cornea in order to obtain a perfect optical parallel. The time from a certain point on the corneal surface to the adjacent point of the laser to the adjacent point of the laser is much longer compared to the cornea, which is more conducive to corneal heat dissipation, and the probability of central island formation is very small. Large cutting light area and good center positioning can effectively reduce surgical complications and improve postoperative predictability [27, 28].

Common operations include: the principle of PRK surgery is that excimer laser is used to cut the central anterior corneal surface after corneal epithelium is scraped, that is, the anterior elastic layer and superficial stroma of the epithelium are removed to reduce the curvature of the anterior corneal surface, thus changing the refractive state of the operative eye [29–31]. Due to the destruction of corneal epithelium and anterior elastic layer during operation, the recovery of postoperative visual acuity was slower compared to LASIK, and the pain was obvious. Subepithelial corneal haze (Haze) appeared after operation, but gradually disappeared within 6 months, and there was no obvious sign under slit lamp examination [29]. LASIK is a surgical method developed on the basis of PRK. Compared with the two, PRK still has its own advantages: There is more room for corneal cutting, thicker corneal bed can be retained after operation, postoperative aberration is small, and there are no complications related to corneal flap. And with the development and maturity of the technology, the shortcomings of the original PRK are greatly reduced. LASIK operation uses automatic micro-lamellar system to make pedicled lamellar corneal flap on the corneal surface. After turning the corneal flap, excimer laser computer is adopted to control multi-step keratectomy. Finally, the corneal flap is restored [32, 33]. This method retains the integrity of corneal epithelium and anterior elastic layer, and excimer laser cutting of the corneal stroma under the corneal flap is mainly through the energy of laser photons to open the chemical bond between tissues, thus producing the cutting effect. Change the curvature of the cornea, and reshape the corneal curvature to correct ametropia. Therefore, the control of corneal thickness is the key to the whole operation. Compared with PRK, LASIK retains the integrity of corneal epithelium and anterior elastic layer, which is more in line with corneal anatomy and physiology. Postoperative infection is rare, there is no pain, visual acuity recovers quickly, no Haze occurs, visual acuity recovers, and refractive state is generally stable within 1-3 months [34]. Its effectiveness and safety have been widely confirmed, but the degree of correction is limited by the thickness of the machinable parenchyma of the cornea [35]. The edge of “C” shaped corneal flap can be seen after operation, and there are some problems related to corneal flap, such as incomplete corneal flap, free corneal flap, and implantation of subflap epithelium [36]. LASEK is a surgical method between PRK and LASIK, which is superior to PRK but cannot replace LASIK. It first makes an epithelial corneal flap, then irradiates it with excimer laser under the flap, and finally restores the epithelial flap. The original upper skin flap fell off within two weeks after operation and was replaced by newly grown epithelium. The deficiency of no epithelium in PRK and the complications of corneal flap in LASIK were effectively solved [37]. Maintain the integrity of the eyeball, with good predictability, stability and safety, a wider range of treatable refraction. More studies have indicated that the visual effect of LASEK is better compared to LASIK, which is another leap of excimer laser correction of ametropia after PRK and LASIK, and provides a new direction for excimer laser correction of ametropia [38, 39]. However, it should be noted that LASEK surgery has two disadvantages: First, the postoperative recovery is slow, which usually takes about a week to restore normal vision; the second disadvantage is that postoperative Haze may appear [40, 41].

At present, most of the criteria for evaluating the efficacy of refractive surgery only use visual acuity and diopter, which cannot explain the blurred vision of some patients in clinical work, although the uncorrected visual acuity is more than 1.0 after operation, especially in cloudy days, at night and poor lighting [42, 43]. Therefore, the evaluation of the efficacy of excimer laser corneal refractive surgery has changed from a single visual acuity and diopter to a comprehensive evaluation of visual quality. Visual quality includes contrast sensitivity, color vision, far and near stereoscopic vision, and low contrast vision [44].

Combined with the results of this study, 9 high-quality literatures were finally included through computer database search, with a total of 4366 samples for meta-analysis. Meta-analysis was performed on the surgical effect of excimer laser corneal refractive surgery, and the results of heterogeneity test indicated that postoperative uncorrected visual acuity. This indicated that there was obvious heterogeneity among the included research data and the combined effect size WMD was analyzed by random effects model. This study found that there was no statistically significant difference in uncorrected visual acuity WMD after excimer laser keratorefractive surgery, indicating that the effect and recovery speed of excimer laser keratorefractive surgery were satisfactory. In this study, there was a statistically significant difference in the WMD of the safety of excimer laser corneal refractive surgery, and the 95% confidence level of the WMD fell below the horizontal line. The right side of the void line, indicating that the excimer laser keratorefractive surgery is safe. The results of this study suggest that the long-term (3 years after surgery) visual quality of excimer laser keratorefractive surgery is considered to be better. The analysis shows that the patients have no obvious pain after excimer laser keratorefractive surgery; the integrity of the corneal elastic layer is maintained; the visual acuity recovers quickly, there is no corneal opacity, long-term use of eye drops is not required, and the postoperative refractive stability is faster. It is easy to retreat and can correct myopia from 1.50 degrees to 10.00 degrees, and the treatment safety is high.

## 5. Conclusion

Excimer laser corneal refractive surgery is effective, safe, fast in recovery and good when treating long-term visual acuity, but more studies and follow-up with higher methodological quality and longer intervention time are needed to further verify it. There are still some things that need to be improved in this paper: The sample size of the included literature is small, which may have a certain impact on the results of the study; the long-term efficacy time of each literature is different, and the combined analysis cannot be carried out, and the safety needs to be further evaluated. Clinically, more large-scale high-quality RCTs are needed to be further verified to provide more reliable evidence-based evidence.

## Figures and Tables

**Figure 1:** Summary of risk of bias. Showing risk of bias as either low (green), unclear (yellow), or high (red) for included studies.

**Figure 2:** Risk of bias assessment of included studies. Showing risk of bias as either low (green), unclear (yellow), or high (red) for included studies, for random sequence generation, allocation concealment, blinding of participants and personnel, blinding of outcome assessment, incomplete outcome data, selective reporting, or other bias.

**Figure 3:** Forest plot of meta-analysis of postoperative uncorrected visual acuity.

**Figure 4:** Forest plot of meta-analysis of preoperative naked visual acuity.

**Figure 5:** Forest plot of meta-analysis of security.

**Figure 6:** Forest plot of meta-analysis of naked eye vision (close).

**Figure 7:** Forest plot of meta-analysis of naked eye vision (far away).

**Figure 8:** Forest plot of meta-analysis of best corrected visual acuity (close).

**Figure 9:** Forest plot of meta-analysis of best corrected visual acuity (distant vision).

**Table 1:** Basic characteristics of literature.

Include the literature	Year of publication	Disease type	Number of samples	Treatment method	Outcome index
Zhao Liankai	2021	High myopia	284/284	Femtosecond laser assisted excimer in situ keratomileusis and lamellar knife flap excimer laser in situ keratomileusis	3, 4
Zheng Xuanbo	2018	Hyperopic anisometropic amblyopia	10	Excimer laser corneal refractive surgery	3, 4, 5, 6
Wang Guofei	2021	Farsightedness and myopia	60/98	Excimer laser corneal refractive surgery	2, 3, 4, 7
Zhang Shengqi	2019	Hyperopic anisometropic amblyopia	43	Excimer laser corneal refractive surgery	3, 4, 5, 6
Gelihua	2018	Farsightedness and myopia	124/52	Excimer laser corneal refractive surgery	1, 2
Liang Caifeng	2018	Farsightedness and myopia	136/50	Excimer laser corneal refractive surgery	1, 2
Guan Yuyan	2018	Hyperopic anisometropic amblyopia	30	Excimer laser corneal refractive surgery	3, 4, 5, 6
Nie Xingang	2017	Hyperopic anisometropic amblyopia	26	Excimer laser corneal refractive surgery	3, 4, 5, 6, 7
Fan Zhengjun	2002	Farsightedness and myopia	3135/34	Excimer laser corneal refractive surgery	1, 2, 7

Note: 1: preoperative naked visual acuity; 2: postoperative uncorrected visual acuity; 3: naked eyesight (close); 4: naked eyesight (farsighted); 5: best corrected visual acuity (close); 6: best corrected visual acuity (vision); 7: security.

## Data Availability

No data were used to support this study.
